# The Efficacy of 18F-FDG PET/CT and Superparamagnetic Nanoferric Oxide MRI in the Diagnosis of Lung Cancer and the Value of 18F-FDG PET/CT in the Prediction of Lymph Node Metastasis

**DOI:** 10.1155/2021/2448782

**Published:** 2021-09-11

**Authors:** Lan Yao, Mingfei Zuo, Na Zhang, Tian Bai, Qicheng Huang

**Affiliations:** ^1^Department of Nuclear Medicine, The Third Affiliated Hospital of Qiqihar Medical University, Qiqihar, Heilongjiang, China; ^2^The Center of Image, The Third Affiliated Hospital of Qiqihar Medical University, Qiqihar, Heilongjiang, China

## Abstract

In China, lung cancer is one of the leading causes of death among residents. Early diagnosis is of great significance for early interventional treatment and prolonging survival. PET/CT uses positron radiopharmaceuticals to observe the physiological and biochemical changes of the drug and its metabolites in the body and finally diagnoses the disease. 18F-FDG is a commonly used imaging agent, but its short isotopic half-life limits clinical high-throughput testing. This study retrospectively analyzed the imaging material of 100 lung cancer patients pathologically confirmed. Patients with lymph node metastasis were classified into the LM group (*n* = 30 cases), and those with no lymph node metastasis were classified into the NLM group (*n* = 70 cases). The results showed that MRI of superparamagnetic nanoferric oxide was better than diagnosis of lung cancer by the 18F-FDG PET/CT and had a high predictive power for lymph node metastasis. These turned out to be high-value lung cancer diagnosis of superparamagnetic nanoferric oxide MRI and high-capacity lymph node metastasis prediction of 18F-FDG PET/CT, which were worthy of implementation.

## 1. Introduction

As a malignant tumor whose primary focus is located in the bronchial mucosal epithelium, lung cancer has the highest mortality and morbidity among cancer diseases, threatening the health and life of patients [1, 2]. Early lung cancer usually has insidious symptoms, and most patients have advanced lung cancer when they are diagnosed, so early diagnosis of lung cancer is very necessary to prolong the survival period for patients to gain treatment time [3]. At present, clinicians mainly make a judgment on lung cancer based on histopathological and imaging examination results, combined with the patient's vital signs and clinical symptoms. Among them, positron emission tomography-computerized tomography (PET-CT) is a common imaging inspection equipment for lung cancer, which integrates PET and CT, dynamically and quantitatively observes the physiological and biochemical changes of positron radiopharmaceutical and its metabolites in the body at the molecular level, is noninvasive, quantifies, and finally diagnoses the disease [4]. However, 18F-FDG is a commonly used metabolic imaging agent labeled by fluorine 18, which can track the metabolic process of glucose in lung tumors, detect the activity and location of lung tumors, and finally make an effective differential diagnosis of lung cancer [5]. Although this diagnostic method is highly sensitive and quantifiable, the short half-life of 18F-FDG isotope limits clinical high-throughput testing, and the presence of 18F-FDG radioactivity can cause toxicity to the patient's organs. Therefore, a sensitive detection method for early diagnosis of lung cancer is still needed. Magnetic resonance imaging (MRI) is a structural image formed by converting the energy released by MRI into electromagnetic waves. Compared with PET, X-ray film, and other imaging technologies, the imaging information provided by MRI has higher clarity and resolution for disease diagnosis [6, 7]. Clinically, contrast agents are used in the process of MRI detection to enhance the contrast effect of images. Conventional contrast agents have a short circulation time in the body, and their biosafety and cytotoxicity are not clear. Superparamagnetic iron oxide nanoparticle (SPION) is a new type of nanomaterial, which has the characteristics of superparamagnetism, good biocompatibility, and targeting [8]. Studies have confirmed that targeted contrast agents with high sensitivity and specificity can significantly improve the diagnostic rate of lung cancer [9]. In addition, lymph node metastasis refers to the phenomenon that tumor cells grow the same tumor after arriving at lymph nodes in the confluence region with lymphatic fluid, which is one of the pathways for tumor cell proliferation [10]. Accurate differential assessment of lung cancer associated with lymph node metastasis can guide the clinician to correspond treatment plan. Therefore, this study also explored the efficacy of N-SUV_max_, T-SUV_max_, T-MTV, T-TLG, and other parameters of 18F-FDG PET/CT in predicting lymph node metastasis, and the data and results of the study were reported in detail below.

## 2. Materials and Methods

### 2.1. Materials

After being approved by the Medical Ethics Committee, patients with primary lung cancer receiving treatment from February 2017 to August 2020 were voted as the subjects of this study. Selection criteria are as follows: (1) in line with clinical diagnostic criteria for lung cancer [11], (2) no treatment prior to 18F-FDG PET/CT and superparamagnetic nanoiron oxide MRI, and (3) complete clinical data. Failing to be chosen criteria are as follows: (1) the presence of coagulation dysfunction or malignant tumor; (2) organic lesions of the heart, liver, and kidney organs; and (3) abnormal hematopoietic function. A total of 100 cases were included. In postoperative paraffin-embedded sections and pathological examination, based on the presence or absence of lymph node metastasis, patients assessed as “yes” were assigned to the LM group (*n* = 30 cases) and those assessed as “no” to the NLM group (*n* = 70 cases).

### 2.2. Method

#### 2.2.1. 18F-FDG PET/CT Examination

The method flowchart is shown in Figure 1. The PET/CT instrument was provided by Huijia Biotechnology (Shanghai) Co., Ltd. 18F was produced by Minitrace accelerator. 18F-FDG comes from tracer lab positron drug synthesis system. Tracer's radiochemical purity was over 95%. On the day examined, after being required to abstain from drinking and fasting for 6 h and to remain fasting with blood glucose level being lower than 7.8 mmol/L, the patients were given intravenous injection of 18F-FDG 4.00-5.50 MBq per kilogram (note that 15 min of rest was required before injection). After maintaining the resting state for 1 h, the patients underwent complete PET/CT examination. Process: the spiral CT scanning parameters were 140 kV tube voltage and 90 mA tube current for scanning, and then, a PET scan was done from the cranioparietal to the superior femur. The CT data were reconstructed by attenuation correction and iterative method and then transmitted to the workstation for image analysis. The tumor metabolism assessment software was opened to analyze PET and CT data. Region of interest (ROI) was drawn for 18F-FDG hypermetabolic tumor lesions, and T-SUV_max_, T-TLG, and T-MTV were obtained. The region of lymph node metabolic abnormality was drawn, and the ROI obtained was N-SUV_max_. Maximum standardisation value (SUV_max_) of 40% of the primary lesion was selected as the threshold; then, all lesions were delineated by ROI technology, SUV_max_ and MTV of primary focus were marked down, and MTV and TLG of ROI were obtained according to the software.

#### 2.2.2. Superparamagnetic Nanoferric Oxide MRI Examination

SPION (provided by Xi'an Ruixi Biotechnology Co., Ltd.) was used as a tracer (Figure 2). The patients' chest was examined using MIR produced by GE in the US. Process: coronal, sagittal, and cross-sectional scans were performed. T1-weighted spin echo imaging was carried out at TR, 583 ms, and TE 15 ms. T2-weighted spin echo imaging was carried out at TR, 4600 ms, and TE 105 ms. The thickness was 5 mm, and T1W1 and T2W1 imaging was obtained. Scanning cross section to coronal plane, select layer thickness of 10 mm and pitch of 1.2 mm. When WB-DWI was positive and MRI was negative, enhanced MRI scan was required. Both images were assessed by 2 seasoned nuclear medicine physicians alone by themselves. Finally, an agreement was reached on the evaluation results.

### 2.3. Indicator for Further Observation

18F-FDG PET/CT detection confirmed criteria: the concentration of mediastinal pool was less than that of the lesion, lobulation sign and burr sign were present at the edge of the lesion, the lesion tissue showed air bronchial sign, thick-walled cavity, ground glass density shadow, etc., and vascular cluster sign and pleural depression sign were present around the lesion [12]. 18F-FDG PET/CT parameters: N-SUV_max_, T-SUV_max_, T-MTV, and T-TLG. Diagnostic criteria of MRI lung cancer: for MRI image score, 1, 2, 3, 4, and 5 represent certainly negative, possibly negative, uncertain, possibly positive, and certainly positive, respectively [13].

### 2.4. Methods of Statistics

SPSS 18.0 software was used to analyze the result data. The measurement data expressed as mean ± standard deviation were compared by *t*-test. Qualitative data represented by percentage of cases were compared by the chi-square test. When the theoretical frequency was between 1 and 4, the chi-square value needed to be corrected. The efficacy of N-SUV_max_, T-SUV _max_, T-MTV, and T-TLG in predicting lymph node metastasis of lung cancer was analyzed by using receiver operating characteristic (ROC) curve. The paired-data McNemar test was executed to compare the specificity and sensitivity. The chi-square value according to the formula is *χ*^2^ = (|*c* − *b*| − 1)^2^/(*c* + *b*),  *c* + *b* ≤ 40. A *P* value less than 0.05 indicates a significant difference.

## 3. Results and Discussion

### 3.1. Diagnostic Efficacy of 18F-FDG PET/CT and Superparamagnetic Nanoferric Oxide MRI in Lung Cancer

For sensitivity, specificity, positive predictive value, negative predictive value, and accuracy, 18F-FDG PET/CT detection for the diagnosis of lung cancer results were 81.97% (50/61), 76.92% (30/39), 84.74% (50/59), 73.17% (30/41), and 80.00% (80/100), respectively (Table 1). Accuracy of superparamagnetic nanoferric oxide MRI detection results were 95.08% (58/61), 97.44% (38/39), 98.31% (58/59), 92.68% (38/41), and 96.00% (96/100), respectively (Table 2).

### 3.2. The Difference of Sensitivity and Specificity between the Two Detection Methods

Compared to 18F-FDG PET/CT detection, superparamagnetic nanoiron oxide MRI detection had higher sensitivity and specificity, with significant differences (*P* < 0.05) (Tables 3 and 4).

### 3.3. Clinical Characteristics of Patients and the Two Groups of 18F-FDG PET/CT Parameters

Compared with the NLM group, the LM group had little difference in gender, age, number of lesions, pathological type, and TNM stage (*P* > 0.05); however, the difference in maximum diameter of lesions and the higher-level N-SUV_max_, T-SUV_max_, T-MTV, and T-TLG did exist (*P* < 0.05, Tables 5 and 6 and Figure 3).

### 3.4. The Prediction Effect of 18F-FDG PET/CT Parameters in Lymph Node Metastasis

In the prediction of lymph node metastasis, the AUC of N-SUV_max_, T-SUV_max_, T-MTV, and T-TLG were 0.717, 0.928, 0.954, and 0.918, respectively. The sensitivity of T-SUV_max_ and T-MTV was higher (90.0% and 93.3%, respectively), and the specificity of the four parameters was all more than 85.0%.

## 4. Discussion

In recent years, the number of patients diagnosed with lung cancer has been high, and the same as morbidity, its mortality is also high and it is a serious tumor. The symptoms of early lung cancer are not obvious. Early detection, early diagnosis, and early treatment are crucial for treatment and prolongation of survival. The gold standard for diagnosis of lung cancer is pathological diagnosis, and imaging examination is the main method for early diagnosis. SPION contrast agent plays an important role in MRI application due to its special superparamagnetic function [14]. In this study, we found superparamagnetic nanoferric oxide MRI and 18F-FDG PET/CT had high value in diagnosis of lung cancer. They could also predict well lymph node metastasis.

On the basis of the data analysis of this study, the sensitivity of 18F-FDG PET/CT and superparamagnetic nanoferric oxide MRI for the assessment of lung cancer was 81.97% and 95.08%, respectively, and the specificity was 76.92% and 97.44%, respectively. Through comparison, the sensitivity and specificity of detection of superparamagnetic nanoferric oxide MRI were significantly higher. This indicated that MRI of superparamagnetic nanoferric oxide was more accurate and effective in the diagnosis of lung cancer. In accordance with the relevant research data, the high diagnostic efficiency of MRI is closely related to imaging with vessels, tracheal foil lymph nodes, and hilar lung [15]. In addition, superparamagnetic nanoferric oxide particles were used as contrast agent for superparamagnetic nanoferric oxide MRI. SPION combines superparamagnetic and nanosized properties. It is not only superparamagnetic but also compatible with human tissues with low toxicity [16, 17]. SPION particle size for the diagnosis of lung cancer is generally 50~100 nm; due to its high affinity with the human reticuloendothelial system, it is easily engulfed by the reticuloendothelial cells on normal lung tissue. The T2-weighted signal of normal lung tissue was reduced and appeared black, while the pathological lung tissue showed no reticuloendothelial cell phagocytosis and no T2-weighted signal change. In this way, the contrast between lung lesions and normal tissues is increased, resulting in improved diagnostic sensitivity and specificity and improved diagnostic efficiency [18–20]. Due to the uneven distribution of superparamagnetic iron oxide nanoparticles in patients, the relaxation rate of superparamagnetic iron oxide nanoparticles is higher and the blood circulation time is prolonged. Therefore, it can push the tissue to dephase in the local magnetic field, resulting in a significant reduction in the transverse relaxation time (T2 value). Finally, the enhanced tissue presents low signal in T2-weighted imaging (T2 WI) and is eventually excreted according to the normal iron metabolism pathway [21, 22]. In lung cancer, the absorption of iron by cancerous cells is significantly different from that of normal cells, and there are significantly more transferrin receptors in cancerous cells [23, 24]. This is because cancerous cells multiply faster, and tissue metabolism speeds up, leading to more new blood vessels. However, due to poor lymphatic reflux within the tumor, iron oxide nanoparticles are easy to pass through the tumor tissue and eventually prolong the retention time (high permeability retention effect), which makes MRI diagnosis of lung cancer more sensitive and specific by superparamagnetic nanoferric oxide, laying a foundation for effective diagnosis and treatment of tumors [25, 26]. The study also showed that there were marked differences in the maximum diameter of lesions between the patients in the two groups. And the markedly higher N-SUV_max_, T-SUV_max_, T-MTV, and T-TLG were in the patients of the LM group. These results suggested that the maximum diameter of the lesion might be one of the causes of lymph node metastasis, and N-SUV_max_, T-SUV_max_, T-MTV, T-TLG, and other parameters might be the result of lymph node metastasis activity. The AUC of N-SUV_max_, T-SUV_max_, T-MTV, and T-TLG in predicting lymph node metastasis were all over 0.7. The sensitivity of T-SUV_max_ and T-MTV was both higher than 90.0 (90.0 and 93.3, respectively), and the specificity of the four parameters was all higher than 85.0. In general, 18F-FDG PET/CT parameters, such as N-SUV_max_, T-SUV_max_, T-MTV, and T-TLG, had high efficacy in predicting lymph node metastasis of lung cancer and could accurately differentiate lymph node metastasis of lung cancer patients, which was basically consistent with relevant research results [27, 28]. Accurate assessment of lymph node metastasis is of great significance for the selection of correct and reasonable treatment plan and prognosis. 18F-FDG PET/CT cannot merely present the morphological changes of pathological tissue but reflect the metabolic information at the molecular level through the changes of parameters such as N-SUV_max_, T-SUV_max_, T-MTV, and T-TLG, which is beneficial for clinicians to carry out preliminary staging and select reasonable treatment plan for lung cancer patients [29, 30]. According to the data, the combined routine examination of 18F-FDG PET/CT can significantly reduce ineffective thoracotomy, effectively reduce exploratory and unnecessary thoracotomy, and reduce patient pain [31]. Therefore, 18F-FDG PET/CT detection to determine lymph node metastasis of lung cancer has positive significance in guiding the clinical treatment plan.

There are some limitations in our study. First, this is a retrospective study, which has the characteristics of some bias. Second, the wide use of superparamagnetic iron oxide nanoparticles cannot be realized now and the safety and efficacy should be further validated.

## 5. Conclusion

SPION contains superparamagnetic iron oxide nanoparticles, and it is an integral part of MRI examination. This study retrospectively analyzed the imaging data, pathologically confirmed lung cancer, and compared the lung cancer diagnosis efficacy of 18F-FDG PET/CT and superparamagnetic nanoferric oxide MRI. It was concluded that superparamagnetic nanoferric oxide MRI could diagnose lung cancer better, and 18F-FDG PET/CT had a high predictive effect on lymph node metastasis. It were indicated that like superparamagnetic nanoferric oxide MRI, 18F-FDG PET/CT had high value in diagnosis of lung cancer. It could also predict well lymph node metastasis.

## Figures and Tables

**Figure 1:** Program flowchart. Lung cancer patients' imaging data were retrospectively analyzed in this study. Patients with lymph node metastasis were classified into the LM group and the NLM group. The diagnosis efficacy of 18F-FDG PET/CT and superparamagnetic nanoferric oxide MRI in lung cancer and the value of 18F-FDG PET/CT in the prediction of lymph node metastasis were analyzed.

**Figure 2:** Superparamagnetic iron oxide nanoparticle (SPION). (a) SPION. SPION has the characteristics of large surface area, biocompatibility, and low coercive force, which create favorable conditions for nuclear magnetic resonance imaging. (b) Electron microscopy figure of SPION. SPION is a nanoscale ferromagnetic molecule, which can be uniformly dispersed in the base carrier liquid. Under the action of external magnetic field, SPION can form a variety of shapes along the magnetic field lines.

**Figure 3:** Relationship between parameters and lymph node metastasis. LM group's N-SUV_max_, T-SUV_max_, T-MTV, and T-TLG were higher.

**Table 1:** Diagnostic efficacy of 18F-FDG PET/CT in lung cancer.

18F-FDG PET/CT	Pathological findings		Total
	+	−	
+	50	9	59
−	11	30	41
Total	61	39	100

*Note*. “+” means positive and “−” means negative.

**Table 2:** Diagnostic efficacy of superparamagnetic nanoferric oxide MRI in lung cancer.

Superparamagnetic nanoferric oxide MRI	Pathological findings		Total
	+	−	
+	58	1	59
−	3	38	41
Total	61	39	100

*Note*. “+” means positive and “−” means negative.

**Table 3:** The difference of sensitivity between the two detection methods.

		18F-FDG PET/CT		Total
+	−			
Superparamagnetic nanoferric oxide MRI	+	48	10	58
	−	2	1	3
Total		50	11	61

*Note*. “+” means positive and “−” means negative. *χ*^2^ = 4.083, *P* = 0.039.

**Table 4:** The difference of specificity between the two detection methods.

		18F-FDG PET/CT		Total
+	−			
Superparamagnetic nanoferric oxide MRI	+	0	1	1
	−	9	29	38
Total		9	30	39

*Note*. “+” means positive and “−” means negative. *χ*^2^ = 4.900, *P* = 0.021.

**Table 5:** Clinical characteristics of patients.

Item	LM group (*n* = 30)	NLM group (*n* = 70)	*χ* ^2^	*P*
Gender			0.578	0.447
Male	20 (32.79)	41 (67.21)		
Female	10 (25.64)	29 (74.36)		
Age (year)			0.002	0.965
<60	14 (29.79)	33 (70.21)		
≥60	16 (30.19)	37 (69.81)		
Number of lesions			0.052	0.819
<10	19 (29.23)	46 (70.77)		
≥10	11 (31.43)	24 (68.57)		
Maximum diameter of lesion (cm)			7.113	0.008
<5.0	8 (17.02)	39 (82.98)		
≥5.0	22 (41.51)	31 (58.49)		
Types of lung cancer			0.846	0.358
Central type	21 (27.63)	55 (72.37)		
Peripheral	9 (37.50)	15 (62.50)		
TNM classification			0.157	0.692
I, II	12 (27.91)	31 (72.09)		
III	18 (31.58)	39 (68.42)		

**Table 6:** Parameter level (*x* ± *s*).

Group	N-SUV_max_	T-SUV_max_	T-MTV (cm^3^)	T-TLG (g)
LM group (*n* = 30)	6.35 ± 1.47	15.64 ± 3.98	23.22 ± 6.15	175.26 ± 48.13
NLM group (*n* = 70)	2.68 ± 0.66	6.03 ± 1.18	12.37 ± 3.28	32.38 ± 8.55
*t*	17.290	18.500	11.480	24.120
*P*	<0.001	<0.001	<0.001	<0.001

## Data Availability

All the raw data could be accessed by contacting the corresponding author if needed.

## References

[1] Norouzi M., Hardy P. (2021). Clinical applications of nanomedicines in lung cancer treatment. *Acta Biomaterialia*.

[2] Zhou F., Qiao M., Zhou C. (2021). The cutting-edge progress of immune-checkpoint blockade in lung cancer. *Cellular & Molecular Immunology*.

[3] Lin J., Zhuo Y., Yin Y., Qiu L., Li X., Lai F. (2021). Methylation of RILP in lung cancer promotes tumor cell proliferation and invasion. *Molecular and Cellular Biochemistry*.

[4] Lutje S., Marinova M., Kutting D., Attenberger U., Essler M., Bundschuh R. A. (2020). Nuclear medicine in SARS-CoV-2 pandemia: 18F-FDG-PET/CT to visualize COVID-19. *Nuklearmedizin*.

[5] Evangelista L., Cuppari L., Menis J. (2019). 18F-FDG PET/CT in non-small-cell lung cancer patients: a potential predictive biomarker of response to immunotherapy. *Nuclear Medicine Communications*.

[6] Li Y., Qiao Y., Chen H. (2018). Characterization of tumor vascular permeability using natural dextrans and CEST MRI. *Magnetic Resonance in Medicine*.

[7] Das S. S., Bharadwaj P., Bilal M. (2020). Stimuli-responsive polymeric nanocarriers for drug delivery, imaging, and theragnosis. *Polymers (Basel)*.

[8] Song X., Yan G., Quan S., Jin E., Quan J., Jin G. (2019). MRI-visible liposome-polyethylenimine complexes for DNA delivery: preparation and evaluation. *Bioscience, Biotechnology, and Biochemistry*.

[9] Zhu L., Zhou Z., Mao H., Yang L. (2017). Magnetic nanoparticles for precision oncology: theranostic magnetic iron oxide nanoparticles for image-guided and targeted cancer therapy. *Nanomedicine (London, England)*.

[10] Sun G., Sun Y., Zou Z., Xu S. (2020). Analysis of segmental lymph node metastasis and clinical features in cT1N0M0 lung adenocarcinoma. *BioMed Research International*.

[11] Aftabi Y., Ansarin K., Shanehbandi D. (2021). Long non-coding RNAs as potential biomarkers in the prognosis and diagnosis of lung cancer: a review and target analysis. *IUBMB Life*.

[12] O’Dwyer E., Halpenny D. F., Ginsberg M. S. (2021). Lung cancer screening in patients with previous malignancy: is this cohort at increased risk for malignancy?. *European Radiology*.

[13] Hu H. (2020). Recent advances of bioresponsive nano-sized contrast agents for ultra-high-field magnetic resonance imaging. *Frontiers in Chemistry*.

[14] Dadfar S. M., Camozzi D., Darguzyte M. (2020). Size-isolation of superparamagnetic iron oxide nanoparticles improves MRI, MPI and hyperthermia performance. *Journal of Nanobiotechnology*.

[15] Zhu W., Xu Y., Jin R., Wu C., Ai H. (2020). MRI tracking of dendritic cells loaded with superparamagnetic iron oxide nanoparticles. *Methods in Molecular Biology*.

[16] Xiao Y., Du J. (2020). Superparamagnetic nanoparticles for biomedical applications. *Journal of Materials Chemistry B*.

[17] Yin J., Yao D., Yin G., Huang Z., Pu X. (2019). Peptide-decorated ultrasmall superparamagnetic nanoparticles as active targeting MRI contrast agents for ovarian tumors. *ACS Applied Materials & Interfaces*.

[18] Reczynska K., Marszalek M., Zarzycki A. (2020). Superparamagnetic iron oxide nanoparticles modified with silica layers as potential agents for lung cancer treatment. *Nanomaterials (Basel)*.

[19] Gkagkanasiou M., Ploussi A., Gazouli M., Efstathopoulos E. P. (2016). USPIO-enhanced MRI neuroimaging: a review. *Journal of Neuroimaging*.

[20] Shen Y., Hu J., Eteer K. (2020). Detecting sub-voxel microvasculature with USPIO-enhanced susceptibility- weighted MRI at 7 T. *Magnetic Resonance Imaging*.

[21] Ugga L., Romeo V., Tedeschi E., Brunetti A., Quarantelli M. (2018). Superparamagnetic iron oxide nanocolloids in MRI studies of neuroinflammation. *Journal of Neuroscience Methods*.

[22] Wei Y., Liao R., Mahmood A. A., Xu H., Zhou Q. (2017). pH-responsive pHLIP (pH low insertion peptide) nanoclusters of superparamagnetic iron oxide nanoparticles as a tumor-selective MRI contrast agent. *Acta Biomaterialia*.

[23] Zhang L., Jin R., Sun R. (2019). Superparamagnetic iron oxide nanoparticles as magnetic resonance imaging contrast agents and induced autophagy response in endothelial progenitor cells. *Journal of Biomedical Nanotechnology*.

[24] Yamaguchi M., Ohnuki K., Hotta K., Fujii H. (2019). MR signal changes in superparamagnetic iron oxide nanoparticle-labeled macrophages in response to X irradiation. *NMR in Biomedicine*.

[25] Can C., Komek H. (2019). Metabolic and volume-based parameters of (18F)FDG PET/CT for primary mass and axillary lymph node metastasis in patients with invasive ductal carcinoma: a retrospective analysis in relation to molecular subtype, axillary lymph node metastasis and immunohistochemistry and inflammatory markers. *Nuclear Medicine Communications*.

[26] Guney I. B., Dalci K., Teke Z. T., Kucuker K. A. (2020). A prospective comparative study of ultrasonography, contrast-enhanced MRI and 18F-FDG PET/CT for preoperative detection of axillary lymph node metastasis in breast cancer patients. *Annali Italiani di Chirurgia*.

[27] Lyu L., Liu Y., Wang X. Y. (2019). Potential value of FDG PET-CT in predicting occult lymph node metastasis in clinical stage IA lung adenocarcinoma. *Zhonghua Zhong Liu Za Zhi*.

[28] Shi Y. M., Niu R., Shao X. L. (2020). Tumor-to-liver standard uptake ratio using fluorine-18 fluorodeoxyglucose positron emission tomography computed tomography effectively predict occult lymph node metastasis of non-small cell lung cancer patients. *Nuclear Medicine Communications*.

[29] Okazaki E., Seura H., Hasegawa Y., Okamura T., Fukuda H. (2019). Prognostic value of the volumetric parameters of dual–time-point18F-FDG PET/CT in non-small cell lung cancer treated with definitive radiation therapy. *AJR. American Journal of Roentgenology*.

[30] Yamamichi T., Kakihana M., Nitta Y. (2020). F-18 fluorodeoxyglucose uptake in lymph nodes and sonographic features on endobronchial ultrasonography predict lymph node metastasis in lung cancer patients. *Journal of Thoracic Disease*.

[31] Sibille L., Seifert R., Avramovic N. (2020). 18F-FDG PET/CT uptake classification in lymphoma and lung cancer by using deep convolutional neural networks. *Radiology*.

